# Role of TLR4/MyD88 Signaling Pathway in the Occurrence and Development of Uremia-Induced Myocardial Hypertrophy and Possible Mechanism

This article has been retracted.

**DOI:** 10.1155/2021/7883643

**Published:** 2021-10-13

**Authors:** Huiping Zhu, Liutong Pan, Yuanting Dai, Dan Zheng, Shasha Cai

**Affiliations:** Department of Nephrology, The First People's Hospital of Wenling, Wenling, Zhejiang 317500, China

## Abstract

The morbidity and mortality of cardiovascular disease (CVD) are relatively high. Studies have shown that most patients with chronic kidney disease (CKD) die from cardiovascular complications. Clinically, the pathophysiological state in which heart disease and kidney disease are causal and influence each other is called cardiorenal syndrome (CRS). Myocardial hypertrophy is the key stage of the heart structure changing from reversible to irreversible. It is an important pathophysiological basis for heart failure. Therefore, this study intends to start with the end-stage uremic phase of CKD to construct an animal model of uremia in rats to study the relationship between uremia, TLR4/MyD88 signaling pathway, and myocardial hypertrophy. The results showed that the uremic rats showed slow weight gain and were thinner. At 12 weeks (w), the serum creatinine and urea nitrogen of the uremic rats increased, and the global hypertrophy index increased. Detecting the expression of Toll-like receptor 4 (TLR4) and myeloid differentiation factor (MyD88) in blood samples of rats, we found that the expression of TLR4 and MyD88 increased at 12 w in the uremia group; pathological observation showed that at 4 weeks of uremia model rats, renal tissue compensatory hypertrophy, renal fibrous membrane proliferation, renal parenchyma atrophy, a large number of fibrous proliferation and inflammatory cell infiltration in the interstitium, and protein casts in the renal tubules were observed. Myocardial cells were obviously hypertrophy and disordered. At 12 w, renal tubules were obviously expanded, the epithelium was flat, the brush border disappeared, and the interstitial fibrous connective tissue of the myocardial tissue was proliferated. The detection of TLR4 and MyD88 in kidney tissue and myocardial tissue revealed that the positive expression of TLR4 and MyD88 gradually increased over time. Therefore, the final result of the study is that uremia can gradually lead to myocardial hypertrophy and TLR4 and MyD88 are highly expressed in serum, kidney, and myocardial tissues of uremic rats, suggesting that TLR4 and MyD88 may be related to the degree of uremic disease and the myocardium caused by it. Hypertrophy is related.

## 1. Introduction

At present, the morbidity and mortality of cardiovascular disease (CVD) have been high and on the rise, especially in patients with chronic kidney disease (CKD), most of which die from cardiovascular complications. The mortality rate of patients with end-stage CKD complicated by CVD is 10–30 times higher than that of the general population [1]. Uremia patients who died of cardiovascular complications accounted for more than 50% of uremia deaths. However, until now, clinicians have generally recognized that cardiovascular events are the leading cause of death in CKD patients. CKD patients often have elevated blood pressure and dyslipidemia [2]. Hypertension and dyslipidemia are the main risk factors for impaired vascular endothelial cell function and the progression of atherosclerosis. Upregulation of inflammatory factors and activation of the renin angiotensin aldosterone system (RAAS) in CKD patients in turn increase the production of reactive oxygen species, accelerate the progression of atherosclerosis, and lead to coronary atherosclerotic heart disease. The incidence of heart failure, stroke, and peripheral arterial disease has increased. In short, CKD increases the incidence and mortality of cardiovascular events, so the prevention and treatment of CVD are particularly important in the management of CKD patients [3].

CKD promotes the impairment of vascular endothelial cell function and the progression of atherosclerosis through various ways and increases the occurrence of cardiovascular events. Conversely, impaired renal vascular endothelial cell function and progression of renal atherosclerosis can also accelerate renal failure. Clinically, the pathophysiological state in which heart disease and kidney disease are causal and influence each other is called cardiorenal syndrome (CRS) [4]. The concept of CRS is helpful to the in-depth study of the pathophysiological mechanism of the interaction between CVD and CKD, to the diagnosis and treatment of patients with CKD and CVD, and to improve the prognosis of patients. Myocardial hypertrophy is the evolution of cardiac function from the compensatory phase to the decompensated phase of heart diseases such as hypertension and valvular disease and the key stage of the change of cardiac structure from reversible to irreversible. It is an important pathophysiological basis for heart failure, but so far the molecular mechanism and cell signal transduction mechanism of myocardial hypertrophy caused by uremia are not yet clear.

Toll-like receptor 4 (TLR4) is the most studied Toll-like receptor; the main ligands are lipopolysaccharide (LPS), respiratory syncytial virus protein, and lipoteichoic acid [5]. TLR4 can activate the transcription and synthesis of inflammatory factors through the myeloid differentiation factor 88 (MyD88) dependent signaling pathway or non-MyD88-dependent signaling pathway and is closely related to the production of inflammatory factors. Wang et al. [6] and other studies found that high glucose can stimulate the increase of TLR4 expression in proximal convoluted renal tubular epithelial cells in mice. Under high glucose environment, the MyD88-dependent TLR4 signaling pathway is activated, indicating that TLR4 is related to inflammation of diabetic nephropathy. Kaur et al. [7] found that the expression of TLR4 and MyD88 in mouse glomerular mesangial cells stimulated by high glucose increased and further promoted the occurrence of diabetic nephropathy. On the other hand, among TLRs, the highest expression in the heart is TLR4 [8]. Studies have found that, in TLR4 knockout mice, the degree of cardiac hypertrophy caused by pressure overload is weakened [9]. The TLR4-mediated MyD88-dependent nuclear factor-*κ*B (NF-*κ*B) pathway is involved in the regulation of cardiac hypertrophy [10]. Blocking MyD88 can reduce the degree of cardiac hypertrophy *in vivo* [11].

In view of this, this study intends to start with the end-stage uremic phase of CKD, construct an animal model of uremia in rats, and study the relationship between uremia, TLR4/MyD88 signaling pathways, and myocardial hypertrophy, which will help to further clarify the myocardium induced by uremia. The pathogenesis of hypertrophy is also beneficial to improve the prevention and treatment of myocardial hypertrophy, thereby effectively reducing the burden on society and families.

## 2. Materials and Methods

### 2.1. Materials and Reagents

Toll-like receptor 4 (TLR4) detection kit (enzyme-linked immunosorbent assay (ELISA)), SEA753Ra, and myeloid differentiation factor (MyD88) detection kit (ELISA), SEB707Ra, were purchased from Wuhan Unison; hematoxylin (SIGMA, article number: H9627, batch number: SLBN3249V); eosin (SIGMA, article number: E6003, batch number: 62R80915X); MyD88 antibody (SANTA company, product number: sc74532, batch number: F2218); TLR4 antibody (Abcam, product number: ab22048, batch number: GR271814); secondary antibody (rabbit kit, Beijing Zhongshan Golden Bridge Biotechnology Co., Ltd., catalog number: PV-6001, batch number: K167722B; mouse kit, Beijing Zhongshan Golden Bridge Biotechnology Co., Ltd., catalog number: PV-6002, batch number: K1566171); automatic biochemical analyzer (Roche Cobas, model: C501); pipette (Beijing Dalong Xingchuang Experimental Instrument Co., Ltd.); full-wavelength microplate reader (SpectraMax Plus 384, USA MD); rotary microtome (RM2235, LEICA company, equipment number: HB215); pathological tissue bleaching and drying instrument (Tec 2500, Changzhou Haosilin Instrument Equipment Co., Ltd., equipment number: HB121); microscope (type BX43, Olympus company, equipment number: HB133); and water-proof constant temperature incubator (type PYX-DHS500BS-II, Shanghai Yuejin Medical Equipment Co., Ltd., equipment number: HB123).

### 2.2. Animal Source

25 male SD rats of SPF grade, weight 200–220 g, were purchased from Shanghai Slack Laboratory Animal Co., Ltd. (license number: SCXK (Shanghai) 2017-0012, certificate number: 03726769). The drinking water used is sterilized secondary ultrapure water. The quality of drinking water meets the requirements of the National Drinking Water Hygiene Standard of the People's Republic of China (GB5749-2006). The license number of the laboratory animal room is SYXK (Zhejiang) 2015-0008. Environment: the temperature range is 20∼25°C, and the relative humidity range is 40∼70%.

### 2.3. Animal Modeling [12]

In this experiment, nephrectomy was used to establish a rat model of uremia to evaluate the effect on the rat's heart. 25 rats were divided into 3 groups: the normal control group (*n* = 6), the mock surgical group (*n* = 6), and the uremia group (*n* = 13). The normal control group did not receive any intervention, and the mock surgical group was only cut. The abdominal cavity was opened without nephrectomy; rats in the uremic group were subjected to 5/6 nephrectomy for modeling. Each group was tested after 4 weeks (w) and 12 w. The rats were anaesthetized and fixed in the supine position. The abdomen was prepared and disinfected and cut along the middle of the abdomen. The right renal blood vessel was separated, the renal vein and renal artery were ligated, and the right kidney was completely removed. The upper and lower poles of the left kidney were each removed 1/3. After hemostasis, the abdomen was closed and 100,000 units of penicillin were injected intramuscularly to prevent infection.

### 2.4. Taking Materials

Three rats were collected at each time. Blood was taken from the abdominal aorta after the rats were anesthetized. The serum was separated at 3500 rpm (8 cm) for 10 minutes to determine the content of urea nitrogen and creatinine in the serum. The expression difference of TLR4 and MyD88 in the serum was detected by ELISA. The heart was weighed, the global hypertrophy index was calculated, and the degree of cardiac hypertrophy was evaluated. Rat kidneys were fixed with 4% formaldehyde for HE staining and immunohistochemistry; hearts were fixed with 4% formaldehyde for HE staining and immunohistochemistry.

#### 2.4.1. Biochemical Testing

After the rats were anesthetized, blood was taken from the abdominal aorta and the serum was separated at 3500 rpm for 10 min. The changes of serum urea nitrogen and creatinine in each group of rats were detected by using an automatic biochemical analyzer.

#### 2.4.2. Determination of Global Hypertrophy Index

The weight of the rat was noted, the rat's thoracic cavity was quickly opened to obtain the heart, the atrium tissue was removed, the surface water was rinsed with saline, and the surface water was absorbed with filter paper. The electronic balance weighed the whole heart to calculate the whole heart weight/body weight, which is recorded as the whole heart hypertrophy index.

#### 2.4.3. ELISA Experiment

ELISA was used to detect the expression of TLR4 and MyD88 in serum. ELISA kits were placed at room temperature for equilibrium, and serum samples were melted at room temperature to avoid repeated freezing and thawing. 50× wash solution was prepared with deionized water as 1× wash solution. 1 ml of standard dilution was added to the standard wells, and the standard dilution was used for gradient dilution. The sample was added and incubated at 37°C for 1 hour. The liquid was discarded and spin dried. Add 100 *μ*L of detection A reagent working solution to each well (prepared immediately before use) and incubate at 37°C for 1 h. Discard the liquid, add 350 *μ*L of 1× washing buffer to each well to wash, soak for 1-2 minutes, and tap the enzyme on absorbent paper. The target plate is to remove all the liquid in the well, and repeat the plate washing 3 times. The washing buffer was poured out after washing, and the remaining liquid was sucked up. 100 *μ*L of detection B working solution (prepared immediately before use) was added to each well and incubated at 37°C for 1 h. The liquid was discarded, dried, and washed 5 times. 90 *μ*L of TMB substrate solution was added to each well and incubated at 37°C 30 min (when the first three standard wells have obvious gradient colors and the last three wells are not obvious, the reaction can be terminated). After ensuring that there were no bubbles and water droplets in each well, use a microplate reader to read statistics at 450 nm.

#### 2.4.4. HE Staining: Sections of Kidney Tissue and Myocardial Tissue Were Made

The tissue was removed from the fixative solution and trimmed to an appropriate shape and thickness; the tissue block was dehydrated by 80%, 90%, 95%, and 100% ethanol I, 100% ethanol II, and 100% ethanol III. The above are the reagents that can be used in the dyeing process. Then, the embedding was carried out and the tissue was embedded in paraffin according to the principle of the material side facing down. After the wax block was cooled and solidified, it was stored at −20°C and refrigerated. Sectioning was done. The thickness was 4 *μ*m. The sections were put in a 65°C thermostat for 6–12 h, dewaxed and rehydrated, immersed in hematoxylin staining solution for 5 min at room temperature, and stained with tap water for 1 min. The sections were immersed in a 1% hydrochloric acid alcohol solution for a few seconds and tap water until the tissue turned blue. Then, the sections were immersed in eosin staining solution for staining. The floating color on the glass slide was removed by washing for 3–5 min with tap water. The above are the reagents that can be used in the dyeing process. The staining results are as follows: the nucleus was blue or purple blue, the cytoplasm was pink, and the red blood cells were bright red. The sample is observed under a microscope, and a comprehensive pathological description of the symptoms of the sample was made.

#### 2.4.5. Immunohistochemistry

Immunohistochemistry was used to detect the positive expression of TLR4 and MyD88 in kidney tissue and myocardial tissue. Kidney tissue sections and myocardial tissue sections were deparaffinized with xylene, rehydrated with gradient alcohol, incubated with 3% H_2_O_2_ at 37°C for 15 minutes, and washed with PBS for 3 × 5 minutes to block and inactivate endogenous peroxidase. Slices were boiled in 0.01 M citrate buffer (pH 6.0) for 10 minutes, cooled to room temperature, and rinsed with PBS for 3 × 5 minutes. The primary antibody (TLR4 (1 : 200) and MyD88 (1 : 75)) was added dropwise, incubated overnight in the refrigerator at 4°C, equilibrated at room temperature for 30 minutes, and rinsed for 3 × 5 min. The secondary antibody was added dropwise, incubated at 37°C for 30 minutes, and washed with PBS for 3 × 5 minutes (PBS was used instead of the primary antibody as a negative control). DAB staining, the progress of the reaction was observed under a microscope, and then fully rinsed with tap water; hematoxylin was counter-stained, then dried, mounted, and photographed. The optical density of MyD88 and TLR4 positive expression was measured with Image-Pro Plus. Five fields of view were measured for each sample, and the final result was expressed as the mean ± standard deviation.

### 2.5. Statistics

The experimental data were expressed as the mean ± standard deviation, and the analysis of variance and statistical test were used the analysis of multigroup means in the GraphPad Prism statistical software. First, the data were tested for the homogeneity of variance; if the variances were uniform, the one-way analysis of variance was used. Statistical methods were used to compare the mean between multiple dose groups and a control group. Data with nonnormality or uneven variance were used for statistics instead of the rank sum test. *P* > 0.05 means that the data are statistically different.

## 3. Results

### 3.1. General Description

A total of 13 uremic rats were modeled, out of which 5 rats died. The dead rats were not included in the statistics, and 8 rats remained in the model group. Uremic rats showed slow weight gain and were thinner.

### 3.2. Changes in Serum Urea Nitrogen and Creatinine in Rats

The results showed that there was no difference in serum creatinine and urea nitrogen levels of rats in each group at 4 w (*P* > 0.05). At 12 w, the serum creatinine and urea nitrogen of rats in the uremia group were higher than those in the normal control group and the mock surgical group and higher than those in the 4 w uremic group, and the difference was statistically significant (*P* > 0.05), as shown in Figures 1(a) and 1(b).

### 3.3. Comparison of Myocardial Hypertrophy Index in Rats

The results showed that there was no statistical difference in the myocardial hypertrophy index of rats in each group at 4 w (*P* > 0.05). At 12 w, the myocardial hypertrophy index of rats in the uremic group was higher than that of the normal control group and the mock surgical group, and the difference was statistically significant (*P* > 0.05), as shown in Figures 2(a) and 2(b).

### 3.4. Observation of Pathological Sections of Rats

The results showed that there were no obvious lesions in the kidney tissue and myocardium in the normal control group and the mock surgical group, but the renal tissue in the 4 w uremia group had compensatory hypertrophy, visible renal fibrous membrane hyperplasia, renal parenchymal atrophy, and a large number of fibers in the interstitium. Hyperplasia, inflammatory cell infiltration, and protein casts can be seen in the renal tubules. Myocardial cells are obviously hypertrophy, and the arrangement is disordered. At 12 w, in the uremia group, the renal tubules are obviously expanded, the epithelium is flat, the brush border disappears, and the interstitial fibrous connective tissue of the myocardial tissue is proliferated. The rest of the lesions are the same as in the 4 w uremia group, as shown in Figure 3.

### 3.5. Expression of TLR4 and MyD88 in Rat Serum

The results showed that the expression levels of TLR4 and MyD88 in the serum of rats in the mock surgical group and the uremia group were higher than those in the normal control group, and the differences were statistically significant (*P* > 0.05). At 4 w, the serum TLR4 level of rats in the uremia group was higher than that of sham operation (*P* > 0.05), but there was no significant difference in the change of MyD88 level (*P* > 0.05). At 12 w, the expression levels of TLR4 and MyD88 in uremic rats were higher than those in the mock surgical group and the 4 w uremic group. The differences were statistically significant (*P* > 0.05), as shown in Figures 4(a) and 4(b).

### 3.6. Expression of TLR4 in Rat Kidney Tissue and Myocardial Tissue

The results showed that, in the kidney tissue, the expression of TLR4 in the uremia group was higher than that in the normal control group and the mock surgical group, and the difference was statistically significant (*P* > 0.05). In myocardial tissue, the TLR4 level of rats in the mock surgical group and the uremia group was higher than that in the normal control group. The TLR4 level of the uremia group was higher than that of the mock surgical group and the level of MyD88 in the uremia group 12 w group was higher than that of the uremia group 4 w group. The differences were statistically significant (*P* > 0.05), as shown in Figures 5(a) and 5(b).

### 3.7. Expression of MyD88 in Rat Kidney Tissue and Myocardial Tissue

The results showed that, in the kidney tissue, the expression level of MyD88 in rats in the mock surgical group and the uremia group was higher than that in the normal control group, the MyD88 level in the uremia group was higher than that in the mock surgical group, and the level of TLR4 in the uremia group 12 w group was higher than that of the uremia group 4 w group. The differences were statistically significant (*P* > 0.05). In myocardial tissue, the MyD88 level of rats in the mock surgical group and the uremia group was higher than that in the normal control group. The MyD88 level in the 12 w uremia group was higher than that in the mock surgical group and 4 w uremia group. The differences were statistically significant (*P* > 0.05), as shown in Figures 6(a) and 6(b).

## 4. Discussion

Uremia is a high-incidence disease in kidney diseases at home and abroad, and research on its symptoms and treatment abounds. However, at present, there are few studies on the molecular mechanism of myocardial hypertrophy as a uremia. The plasma catecholamine concentration increases during uremia, and its degree of increase is closely related to the occurrence of heart failure. In addition, high blood pressure accelerates the progress of atherosclerosis and promotes heart failure [13]. This study explored the mechanism of myocardial hypertrophy in uremia by establishing uremia model rats. Detection of the serum urea nitrogen and creatinine showed that the urea nitrogen and creatinine of the uremic model rats increased significantly at 12 w. In uremic model rats, at 4 w, renal tissue hypertrophy, renal fibrous membrane proliferation, renal parenchyma atrophy, a large number of fibrous proliferation and inflammatory cell infiltration in the interstitium, and protein casts in the renal tubules were observed. At 12 weeks, the tubules were obviously expanded, the epithelium was flat, and the brush border disappeared. The above results indicate the successful establishment of a mouse model of uremia. We observed the heart of model rats and found that the global hypertrophy index of model group rats was higher than that of sham operation and normal group rats. At 12 w, myocardial cells were obviously hypertrophy and arranged disorderly. Myocardial tissue interstitial fibers and connective tissue proliferated significantly, indicating uremia symptoms have the risk of causing myocardial hypertrophy. Myocardial hypertrophy often causes CVD such as heart failure, stroke, and peripheral artery disease and increases the mortality rate. Therefore, the prevention and treatment of CVD are of great significance in the treatment of CKD patients.

In recent years, the role of TLRs in the pathogenesis of kidney disease has received increasing attention. Among them, TLR4 is a type I transmembrane receptor encoded by endotoxin, which is mainly expressed on endothelial cells, epithelial cells, macrophages, and neutrophils. Research reports [14, 15] have shown that TLR4 has two signaling pathways: MyD88-dependent signaling pathways and non-MyD88-dependent signaling pathways. The combination of TLR4 and MyD88 is the earliest event that occurs during the activation of MyD88-dependent signaling pathways. Trentin-Sonoda et al. [16] found that the TLR4/MyD88 signaling pathway played a key role in the evolution of renal ischemia-reperfusion injury from acute renal failure to chronic renal failure.

In our study, the detection of the expression of TLR4 and MyD88 in rat blood samples found that the expression of TLR4 and MyD88 in the uremia group increased significantly at 12 w. The detection of TLR4 and MyD88 in kidney tissue and myocardial tissue revealed that the positive expression of TLR4 and MyD88 gradually increased over time. This may be because in the process of progressive renal fibrosis, due to the increase of matrix, the endogenous ligand exposure of TLR4 on macrophages increases, such as heat shock protein 60, fibrinogen, heparin sulfate, fibronectin EDA, and hyaluronic acid. Endogenous ligands can activate TLR4. Activated TLR4 and related ligands induce NF-*κ*B activation, initiating the transcription of interleukin-1, interleukin-6, interleukin-8, interleukin-12, tumor necrosis factor-*α*, and CD80 and CD86 genes and mediating the recognition and immune activation of various pathogens, resulting in kidney damage [17–19]. In the MyD88-dependent signaling pathway, after TLR4 recognizes and binds to the pathogen-associated molecular pattern (PAMP), it binds to MyD88 through its TIR region (Toll/IL-1 receptor domain) and activates the interleukin-1 receptor associated kinases (IRAK), tumor necrosis factor receptor associated factor 6 (TRAF6), complex membrane protein transforming growth factor related kinase 1 (TAK1), I*κ*B kinase (IKK), and a series of proteases, which lead to the activation of NF-*κ*B translocation to the nucleus and start tumor necrosis factor (TNF)-*α* and other inflammatory factors gene expression [20–22]. This study also observed that compared with the normal control group, the levels of TLR4 and MyD88 were increased in the sham operation group, which may be related to the transcription of inflammatory factors, etc. in the sham operation group, as mentioned above. Rats in the sham operation group underwent open surgery. It is possible that the level of inflammatory factors in the body will be upregulated, leading to an increase in the levels of TLR4 and MyD88.

## 5. Conclusion

In summary, the final result of the study shows that uremia can gradually lead to myocardial hypertrophy and TLR4 and MyD88 are highly expressed in serum, kidney, and myocardial tissues of uremic rats, suggesting that TLR4 and MyD88 may be related to the degree of uremia and the degree of disease caused by it. Myocardial hypertrophy is related. This study can provide an experimental basis for the theoretical research system of the molecular mechanism of uremia-induced myocardial hypertrophy. However, because of time and funding issues, the specific regulatory mechanism of TLR4 and MyD88 has not been studied. Therefore, in-depth study of the specific regulation or regulatory mechanism of the TLR4/MyD88 signaling pathway in the development of uremic myocardial hypertrophy can further explore the level of diagnosis and treatment of uremia and its complications and the level of theoretical research.

## Figures and Tables

**Figure 1:** Changes of urea nitrogen and creatinine in serum of rats. Note: compared with the normal control group at the same time point, ^*∗*^*P* > 0.05; compared with the mock surgical group at the same time point, ^#^*P* > 0.05; and compared with the 4 w uremia group, ^+^*P* > 0.05.

**Figure 2:** Comparison of myocardial hypertrophy index in rats. Note: compared with the normal control group at the same time point, ^*∗*^*P* > 0.05; and compared with the mock surgical group at the same time point, ^#^*P* > 0.05.

**Figure 3:** Observation of pathological sections of rats (100×). Note: the black arrow indicates the infiltration of inflammatory cells, the red arrow indicates the protein cast, and the blue arrow indicates the fibrosis.

**Figure 4:** Expression of TLR4 and MyD88 in rat serum. Note: compared with the normal control group at the same time point, ^*∗*^*P* > 0.05; compared with the mock surgical group at the same time point, ^#^*P* > 0.05; and compared with the 4 w uremia group, ^+^*P* > 0.05.

**Figure 5:** Expression of TLR4 in rat kidney tissue and myocardial tissue (100×). Note: compared with the normal control group at the same time point, ^*∗*^*P* > 0.05; compared with the mock surgical group at the same time point, ^#^*P* > 0.05; and compared with the 4 w uremia group, ^+^*P* > 0.05.

**Figure 6:** Expression of MyD88 in rat kidney tissue and myocardial tissue (100×). Note: compared with the normal control group at the same time point, ^*∗*^*P* > 0.05; compared with the mock surgical group at the same time point, ^#^*P* > 0.05; and compared with the 4 w uremia group, ^+^*P* > 0.05.

## Data Availability

The data used during the current study are available from the corresponding author.
